This article has been retracted.

# Evaluation of the safety of retroperitoneal laparoscopic partial nephrectomy by investigating the perioperative indicators

**DOI:** 10.3389/fonc.2023.1138210

**Published:** 2023-04-19

**Authors:** Xiaoyan Zhang, TianJun Xing

**Affiliations:** ^1^Department of Radiology, Shanxi Bethune Hospital, Taiyuan, China; ^2^Urology Surgery, Shanxi Cancer Hospital, Taiyuan, China

**Keywords:** CT imaging, residual renal function, partial resection of renal cell carcinoma, renal cell carcinoma, RLPN

## Abstract

**Background:**

In recent years, open nephron sparing partial nephrectomy (OPN) has been gradually applied and generally accepted. Recent statistical data show that PN not only can safely and effectively preserve the functional nephron, but also has fewer complications, low local recurrence rate and no significant difference in long-term survival rate compared with nephrectomy/radical nephrectomy, which has gradually become a routine treatment for small renal cell carcinoma. Therefore, how to maximize the protection of postoperative residual renal function (RRF) and reduce the risk of CKD while achieving the ideal local and overall tumor control effect is the key to the treatment of renal cancer, and is also the focus of attention of urologists and nephrologists.

**Objective:**

To evaluate the safety of retroperitoneal laparoscopic partial nephrectomy (RLPN) by investigating the perioperative indicators and postoperative follow-up.

**Methods:**

A total of 40 hospitalized patients in our hospital from December 2019 to December 2021 were selected and followed up for a long time. Patients with renal tumors less than 4cm in diameter and exogeneous or partial exogeneity were randomly divided into 2 groups. Patients in retroperitoneal laparoscopic group (n = 20) were treated with nephron sparing partial nephrectomy (0.5-1cm). Twenty patients underwent retroperitoneal laparoscopic radical nephrectomy (LRN).The time of removal of drainage tube, drainage volume, time of feeding activity and postoperative hospital stay were recorded, and the safety of the operation was evaluated.

**Results:**

nephron sparing partial nephrectomy is suitable for patients with localized renal carcinoma or benign tumor <4cm. RLPN can be applied to all indications of open nephron sparing partial nephrectomy (OPN), with good safety, and can preserve residual renal function to the greatest extent. The operative vascular occlusion time was controlled within 40 minutes, and the use of renal function protection measures during the operation was safe and controllable in reducing the prevention of warm ischemic kidney damage, with good safety. The renal tumor capsule with 0.5cm~1cm margin was complete by postoperative pathology. In the process of tumor resection and suture collection system in the RLPN group, we improved the previous operation of “resection before hemostasis” to “resection while hemostasis” and “knot-free suture” technology, which saved the operation time of intracavity suture knotting. Reduced cortical tear caused by vertical pull during knot tying. The combined effect of biological clip and hemostatic gauze can stimulate the granulation proliferation of renal cortical wound and accelerate the repair. With the combination of knot-free suture and renal segment vascular occlusion, hot ischemic kidney damage is reduced. In the RLPN group, there were no complications of urinary fistula and bleeding, and no abnormal changes in renal function during follow-up. The safety of RLPN group is worthy of affirmation.

**Conclusion:**

The perioperative safety and short-term postoperative renal function recovery of RLPN are good, and the overall safety of this operation is worthy of affirmation.

## 1 Introduction

Renal cell carcinoma, also known as renal cell carcinoma, originates from tubular epithelial cells of the kidney and is the most common malignant tumor of the renal parenchyma (1–3). Renal cell carcinoma has the highest mortality rate among genitourinary tumors (1–3). The vast majority of renal cell carcinomas occur in the unilateral kidney, often a single tumor, and 10% - 20% are multiple lesions, which are common in patients with hereditary renal cell carcinoma and renal papillary adenocarcinoma. Most of the tumors are located at the upper and lower poles of the kidney, and the tumor body is quite different. There is often a pseudocapsule separated from the surrounding renal tissue. In recent years, with the rapid development of medical imaging technology and the aggravation of population aging, the incidence of renal cell carcinoma has increased significantly, and it has become one of the common malignant tumors in developed countries. According to the National Cancer Institute of the United States, there were about 65,340 new cases of renal cancer in the United States in 2018, accounting for about 3.8% of new tumors (3–7).

With the popularization of B-mode ultrasound, computed tomography (CT), magnetic resonance imaging (MRI) and other imaging examinations, the early diagnosis of small renal cell carcinoma has been improved, and the timing of surgical intervention has been advanced (8–10). Traditional radical nephrectomy (RN) may affect renal function due to the removal of one kidney, especially solitary renal cell carcinoma, bilateral renal cell carcinoma, and renal cell carcinoma with contralateral renal damage (8–10). In recent years, open nephron sparing partial nephrectomy (OPN) has been gradually applied and generally accepted (8–10). Recent statistical data show that PN not only can safely and effectively preserve the functional nephron, but also has fewer complications, low local recurrence rate and no significant difference in long-term survival rate compared with nephrectomy/radical nephrectomy, which has gradually become a routine treatment for small renal cell carcinoma (8–10).

Surgical resection remains the first choice for most patients with renal cancer, including radical nephrectomy (RN) and partial nephrectomy (PN). Due to the sharp reduction of renal function units after surgery, the risk of new or progressive chronic kidney disease (CKD) after surgery increases (8–10). Studies have confirmed that CKD is an independent risk factor for cardiovascular disease, hospitalization and death, and is a global public health problem (11–13). How to maximize the protection of postoperative residual renal function (RRF) and reduce the risk of CKD while achieving the ideal local and overall tumor control effect is the key to the treatment of renal cancer and is also the focus of attention of urologists and nephrologists. Therefore, this study evaluated residual renal function after partial nephrectomy based on CT imaging. The purpose of this paper is to investigate the perioperative indexes and postoperative follow-up of retroperitoneal laparoscopic partial nephrectomy (RLPN), and to evaluate its safety.

## 2 Methods

### 2.1 Participants

Patients hospitalized in our hospital from December 2019 to December 2021 were selected for long-term follow-up and complete clinical data were collected. Informed consent was obtained from the patients and the informed consent was signed, which met the ethical requirements of our hospital.

Inclusion criteria: (1) Single tumor; (2) Diameter < 4 cm; (3) Exogeneity or partial exogeneity of the tumor; (4) CT/MR and other imaging examinations did not indicate distant metastasis, and the lesions were localized; (5) Preoperative SCr < or less 300 μmol/L.

Exclusion criteria: (1) There are contraindications for surgery; (2) The preoperative SCr > 300 μmol/L; (3) Severe bleeding tendency; (4) The lesion invaded the renal pelvis or hematuria.

### 2.2 Clinical data

From 2019 to 2021, 20 patients underwent retroperitoneal laparoscopic partial nephrectomy (RLPN). Imaging examination showed isolated renal mass, which was partially exoplasmic, with diameters <4cm, and no signs of renal pelvis or surrounding invasion. Contralateral renal function was normal. Laboratory tests, chest radiograph and other preoperative evaluations did not indicate concomitant surgery. All 20 patients were followed up for 6 months to 2 years, and renal function was reexamined.

### 2.3 Surgical method

Small incisions were made under the costal margin of the posterior axillary line, 2cm above the iliac crest of the midaxillary line and under the costal margin of the anterior axillary line, and three cannulas were placed. The retroperitoneal space was separated by finger or self-made air bag expansion, and the pneumoperitoneum machine was connected. The pressure was set at 15mmHg, and the laparoscope was entered. The renal artery was dissociated and not blocked. Free renal tumor and 2 cm of surrounding kidney. Inosine 2 g was dropped quickly. The renal artery was blocked. Tumor resection: The renal tumor and its marginal renal tissue were removed with ultrasonic knife or scissors. During the cutting process, the absorbable biological clip was used to clamp the cortex along the cut edge with rich blood supply to block the blood vessels in the renal segment. After the tumor was completely removed, the hemostatic effect on the wound could be achieved to a large extent. When the collecting system was closed with 3-0 micro-jotting thread, a biological clip was first put on the end of the thread at the needle inlet, and the cortex was sutured with figure-of 8 suture. At the end of the thread at the needle outlet, a biological clip was used to tighten the end of the thread close to the cortex, and the wound was closed by fixing the two clips. The wound was then covered with hemostatic gauze and sprayed with biological protein glue. The margin tissue was cut and sent for pathological biopsy. Wound vessels were hemostatic by suture with ultrasonic knife combined with absorbable suture, renal pelvis and calyces were sutured with absorbable suture, the wound was stuffed with hemostatic gauze and other materials, and the renal parenchyma wound was sutured initiatively with 2-0 absorbable figure-of 8 suture. The renal artery was opened, and the wound was further sutured to stop bleeding. The drainage tube was placed, the cannula was withdrawn, and the incision was sutured.

### 2.4 Observational index

Drainage related indicators, Postoperative recovery of the patient, Liver function evaluation index were recorded in the group. RLPN patients were followed up 3 months after operation for CT examination and creatinine to understand renal function. The local recurrence rate and survival rate of tumor were studied by follow-up for more than half a year.

All participants were asked to fast for at least 12 hours before taking a venous blood sample. After professional training, nurses use disposable blood needle, strictly follow the standard of aseptic blood collection, morning collection of fasting venous blood 3ml. SCR was measured by standard laboratory procedures and calculation of GFR by the Cockcroft-Gault equation using age, weight and sex, formula=(140-age) x Weight in kg x (0.85 if female)/72 x Cr).

### 2.5 Statistical method

The comparison between the data of two groups was determined with the *t* test, data of the paired two groups were examined by the paired *t* test, and the unpaired student’s *t* test was carried out to compare the differences between the two groups. The Tukey-Kramer test was used for one-way ANOVA on multiple sets of data. SPSS20.0 (SPSS Inc., Chicago, Illinois, USA) was employed to calculate the mean ± SEM results in the experiment. The GraphPad Prism software (version 8.0) was applied for drawing. The difference had statistical significance when *P*<0.05.

## 3 Results

### 3.1 The general information

All the patients were operated smoothly. None of the RLPN patients was transferred to open. None of the RLPN patients received blood transfusion during the operation. None of the patients had complications such as urinary fistula after the operation. Postoperative pathological results: papillary renal cell carcinoma in 1 case (5.0%), clear cell carcinoma in 17 cases (85.0%), spindle cell carcinoma in 2 cases (10.0%); The pathological report after operation showed that the margin was not positive, and the capsule was complete. The closest distance between the margin and the capsule was 0.3cm for a clear cell carcinoma in the RLPN group. The follow-up period ranged from 6 months to 2 years. The follow-up rate was 100%, and the average follow-up period was 14.25 months. From December 2019 to December 2021, 20 patients were in the RLPN group, including 12 males and 8 females, ranging in age from 35 to 67 years (mean age 45.61 ± 4.42 years). In the LRN group, there were 20 patients (10 males and 10 females), ranging in age from 37 to 64 years (mean age 46.42 ± 5.62 years). According to Warren AY et al, renal cell carcinoma is classified into 3 types: spindle cell carcinoma, clear cell carcinoma, papillary renal cell carcinoma, and cell carcinoma (14). There was no complication such as postoperative hemorrhage and urinary fistula, or recurrence and metastasis of malignant tumor in **Table 1**.

**Table 1:** Analysis of baseline data.

Baseline information	RLPN group n	LRN group n	*P* value
Total	20	20	
Gender			0.525
Male	1 2	10	
Female	8	10	
Age	45.61±4.42	46.42±5.62	0.605
≤60	8	9	0.773
>60	12	11	
Papillary renal cell carcinoma/case	1	2	
clear cell carcinoma/case	17	16	
spindle cell carcinoma/case	2	2	
The follow-up	6 months to 2 years	6 months to 2 years	
The follow-up rate/%	100	100	
The average follow-up period/month	14.25	15.32	

### 3.2 Drainage related indicators

The drainage volume and drainage time of RLPN are shown in **Table 2**. The results showed that there was no significant difference in drainage volume and drainage time between RLPN group and LRN Group (**Table 2**; **Figure 1**, *P*>0.05).

**Table 2:** The Drainage related indicators.

Group	Number	Drainage volume/mL	Drainage time/min
RLPN	20	60.27 ± 6.67	3.04 ± 0.35
LRN	20	57.66 ± 5.23	3.22 ± 0.43
*P* Value		0.165	0.144

**Figure 1:** Statistical chart of the difference between Drainage volume **(A)** and indicators **(B)** between the two groups of patients.

### 3.3 Postoperative recovery of the patient

The time to recovery of postoperative bowel function and length of hospital stay were used as criteria for evaluating surgical outcomes. The results showed that compared with the LRN group, patients in the RLPN group had shorter gastrointestinal recovery times and shorter hospital stays than those in the LRN group (*P*<0.05, **Table 3**).

**Table 3:** The postoperative recovery of the patient.

Group	Number	Intestinal recovery time/day	Postoperative hospital stay/day
RLPN	20	2.51 ± 0.48	8.33 ± 1.20
LRN	20	2.87 ± 0.56	10.23 ± 1.42
*P* Value		0.03	<0.001

### 3.4 Liver function evaluation index

SCr and GFR were reexamined 3 months after operation, The renal function was improved after operation as compared with that before operation, which showed a decrease in SCR and an increase in GFR (**Table 4**; **Figure 2**). In addition, we examined the expression of SCR and GFR between the RLPN group and the LRN group at 3 months postoperatively, and the results showed that SCR was decreased and GFR was increased in the RLPN group compared with the LRN Group (*P*<0.05,**Table 5**).

**Table 4:** The liver function evaluation of the patient.

Index	Number	Time	Content (μmol/L)
SCr	20	preoperative	178.33 ± 7.57
		postoperation	110.32 ± 11.26
GFR	20	preoperative	46.82 ± 4.34
		postoperation	71.33 ± 7.40

**Figure 2:** The level of SCR **(A)** and GFR **(B)** in the RLPN group.

**Table 5:** SCR and GFR comparison between RLPN group and LRN Group.

Group	Number	SCr(μmol/ml)	GFR(mL/min)
RLPN	20	110.32 ± 11.26	71.33 ± 7.40
LRN	20	132.33 ± 11.33	57.33 ± 6.24
*P* Value		<0.001	<0.001

## 5 Discussion

Surgical resection is the first choice of treatment for localized renal Cancer, including RN and PN. The specific protocol is mainly based on the International Union against Cancer and the American Joint Committee on Cancer (AJCC) the 8th edition of the TNM staging system for renal cancer implemented in 2018 (15). Early RN is recognized as the standard treatment for localized renal cancer, while PN is only used to treat patients with solitary renal cancer, bilateral renal cancer, or contralateral renal insufficiency (16–21).

In recent years, with the development of medical imaging technology and the improvement of people’s health awareness, the diagnosis rate of early renal cancer has increased significantly. In view of the increasing maturity of surgical techniques, the 5-year survival rate of T1 renal cell carcinoma is over 90% and T1a renal cell carcinoma is close to 100% (22–24). However, the incidence of postoperative CKD is still high, and studies have found that T1 renal cancer patients are more likely to die of CKD-related complications than tumor-related complications (25–27). Therefore, the treatment of early renal cell carcinoma began to change to the direction of preserving renal function, and the clinical application of PN gradually increased.

Currently, retain the nephron renal resection by open surgery to minimally invasive surgery way after laparoscopic technique, both the operation principle is consistent in theory, the safety of OPN and accreditation has been widely, but in RLPN operation safety study, clinical workers are still operating under the cavity mirror details did not form a unified opinion, Such as the grasp of RLPN surgical indications, methods of intraoperative blood vessel blocking, warm ischemia time control, intraoperative renal protection measures, collection system shutdown method and postoperative renal function recovery and other security is still in doubt, in view of the above problem, this study will be emerging RLPN and mature OPN perioperative indicators of comparison, to evaluate the security of the former (28, 29).

At present, its indication is single exoplasmic tumor <4cm, but the relative indication can be relaxed to < 7cm^3^ (30). In this study, the average tumor volume of the RLPN group was 3.46cm, all within the indicated range, and the postoperative efficacy was good. In terms of the choice of surgical methods, RLPN could be basically applicable to all indications of OPN, and the operation safety was good. In the actual operation process, the tumors located in the upper pole of the difficulty of processing than lower pole position is complex, the reason is that tumors had been more than 11 rib intercostals organization cover have led to the exposure of operative field harder, but RLPN group in the imaging system of amplification effect, did not differ by tumor location and increase operation difficulty of operative field, Especially in the intercostal tissue covering factors above 11 ribs, it is not affected, and can achieve a more precise hemostatic effect.

In terms of the comparative study on the time of vascular occlusion, some studies believe that the hot ischemia time <30min has little damage to renal function, while other scholars believe that the limit of blocking time should be controlled within 40 min (1, 31, 32). In this study, the operative vascular occlusion time of patients was controlled within 40min, and renal function protection measures were applied during the operation. In the prevention of reducing hot ischemic kidney damage, the safety is good within a safe and controllable time. According to the comparison data of sCr and GFR changes of patients before and after surgery, there was no difference due to the different surgical methods. It was found that the GFR of the affected kidney decreased slightly after surgery, and there was no statistical difference in the preoperative and postoperative changes, suggesting the safety of long-term recovery after surgery. RLPN can achieve the efficacy of OPN, and it is safe and reliable.

At present, there is still a lot of controversy on the definition of surgical margin. The previous view is that benign tumors can be resected close to the capsule, while malignant tumors need to be resected 1cm away. Some scholars do not advocate the margin of more than 1cm, and believe that the margin can be reduced to less than 1cm to maximize the preservation of nephron function (33, 34). After blocking the blood vessels, we used the ultrasound knife to pre-label the surgical margin in the normal tissue 0.5cm~1cm away from the surrounding tumor, and there was no significant difference in the technical difficulty of surgical resection. According to the postoperative pathological report, the renal tumor capsule of the two groups was complete, which may suggest that the 0.5cm surgical margin can be used as the limit surgical margin selection for renal tumors of uncertain nature. And it has safe operability. Considering the small number of this study group and the lack of quantitative grouping of tumor resection margins, the conclusion of safe resection margin is still particularly limited and needs to be supported by large sample clinical trials. However, for the selection of resection margins for malignant tumors, the authors believe that 0.5cm resection margin is still safe range for malignant tumors.

In the process of surgical resection of tumor body and suture collection system in RLPN group, we improved the previous operation of “resection before hemostasis” and changed it to “hemostasis while resection” and “knot free suture”. In the process of ultrasonic knife cutting, absorbable biological clips are used to clamp the cortex along the incision at the cortical part of the cutting edge with abundant blood supply. After complete resection of the tumor body, the hemostatic effect on the wound can be achieved to a large extent at the same time; When closing the collection system with 3-0 micro Joe, first put a biological clamp on the thread tail at the needle inlet, and then suture the cortex in “8” shape in full layer. At the thread tail at the needle outlet, tighten the thread tail with a biological clamp and glue. The wound is closed by fixing the two clamps. Then, the wound is covered with blood stopping gauze and sprayed with biological protein glue. After opening the renal pedicle, good hemostatic effect is obtained. The advantage of this method is that it saves the operation time of suture knot in the cavity; It reduces the cortical tear caused by vertical pulling during knotting; The combination of biological clamp and hemostatic gauze can stimulate granulation proliferation of renal cortex wound and accelerate the repair (35); In addition, with the use of this knot free suture technique, the renal pedicle blocking time in the late stage of RLPN group can be shortened by about 5-6 minutes compared with that in the early stage, which greatly reduces the renal damage caused by thermal ischemia. There were no complications of urinary fistula and bleeding after operation. The renal function was well changed during follow-up, and the safety was worth affirming.

## 6 Conclusions

RLPN can preserve renal function to the greatest extent on the basis of complete tumor resection, and minimize the trauma to patients. It has good perioperative safety and short-term postoperative renal function recovery. It is safe and reliable, and worthy of wide application.

## Data availability statement

The original contributions presented in the study are included in the article/supplementary material. Further inquiries can be directed to the corresponding author.

## Ethics statement

The study was approved by the hospital’s ethics committee. The patients/participants provided their written informed consent to participate in this study. Written informed consent was obtained from the individual(s) for the publication of any potentially identifiable images or data included in this article.

## Author contributions

XZ were major contributors in writing the manuscript. TX did literature searches, and revised the manuscript. All authors read and approved the final manuscript. All authors contributed to the article and approved the submitted version.
